# Nation Binding: How Public Service Broadcasting Mitigates Political Selective Exposure

**DOI:** 10.1371/journal.pone.0155112

**Published:** 2016-05-24

**Authors:** Linda Bos, Sanne Kruikemeier, Claes de Vreese

**Affiliations:** Amsterdam School of Communication Research ASCoR, University of Amsterdam, Amsterdam, The Netherlands; National Scientific and Technical Research Council (CONICET)., ARGENTINA

## Abstract

Recent research suggests that more and more citizens select news and information that is congruent with their existing political preferences. This increase in political selective exposure (PSE) has allegedly led to an increase in polarization. The vast majority of studies stem from the US case with a particular media and political system. We contend that there are good reasons to believe PSE is less prevalent in other systems. We test this using latent profile analysis with national survey data from the Netherlands (n = 2,833). We identify four types of media use profiles and indeed only find partial evidence of PSE. In particular, we find that public broadcasting news cross-cuts all cleavages. This research note offers an important antidote in what is considered a universal phenomenon. We do find, however, a relatively large segment of citizens opting out of news consumption despite the readily available news in today’s media landscape.

## Introduction

The last decade has produced overwhelming popular and scientific evidence of selective exposure to political messages. According to this strand of research, citizens (carefully) select only messages that are in line with their already existing political preferences and avoid news content based on anticipated disagreement. This process of ‘political selective exposure’ (PSE) has been found to produce a range of undesired outcomes such as polarization, attitude extremity, incivility, and lack of understanding for opposing points of views (for an overview of the literature, see [1]). Recent years’ developments in the media landscape have augmented these processes and made it increasingly easy to self-select a media diet consonant with existing views. The vast majority of this research is based on observations in the United States, which has both a political and a media system that–at least comparatively speaking–cater to such dynamics.

In this research note we take a step back and ask a simple, but fundamental question: to what extent do we find traces of PSE in a non-US context which is rather dominated by a multiplicity of political parties and a different configuration of the media system? Even in the US literature there is disagreement with regard to the extent of PSE and scope of the negative consequences (see [2] [3]). We posit that in a system characterized by more choice on the supply side of politics, less historical roots for polarization, and a media system with less political parallelism, we should address first things first and assess the extent and conditions under which PSE might take place before jumping on the ‘academic bandwagon’ and immediately assess all kinds of (un)desired effects of PSE. In that respect it is rather striking how little research outside the US context on the nature and extent of PSE is found. This is exactly the purpose of our Research Note.

In this Research Note we will focus on the Dutch case to assess the extent of PSE, i.e., the situation in which partisans expose themselves to certain news content, based on anticipated alignment between their attitudes and the content, and avoid other news content, based on anticipated *dis*agreement. Using latent profile analysis with national survey data (n = 2,833), tapping individual exposure (i.e. the consumption of different media) to a large variety of media sources, we identify four types of media use profiles. Our findings show that there are indeed different groups in society with distinctive media diets which is indicative of selective exposure. First of all, we lay out the character of these four profiles in order to tease out the differences and similarities in media preferences between them. Secondly, to understand whether this selective exposure is also *political* in nature, we estimate the impact of partisan preferences on profile membership, controlling for alternative explanations.

## Theory

### Political Selective Exposure

The tendency of media consumers to select information that is in line with their predispositions is not new (e.g., [4] [5] [6]). Indeed, in the US and beyond, the partisan press and close relationships between politics and media organizations, often dubbed as ‘press-politics parallelism’ ([7]) are historically well-documented phenomena. However, recent evidence suggests that there is a resurgence in PSE in a sense that citizens both more and more ascribe (perceived) political positions to media organizations and outlets and increasingly select and process news and information based on (perceived) political preference congruence ([2] [8]). Though the evidence seems pervasive in the US context, there are good reasons to question certain assumptions and be cautious about the universality and ‘direct import’ of US generated concepts (see e.g., [9]).

### Consequences of Political Selective Exposure

Why should we care about PSE? PSE contributes to a polarization of political attitudes ([10]), increases ideological homogeneity ([11]), and changes the way partisans react to threats ([12]). Iyengar and Westwood ([13]) even suggest that–in part through selective media exposure–the level of fear and loathing across political party lines is now much stronger in the past and much stronger than other cleavages such as religion, education, or ethnicity.

#### Questioning the ‘obvious’

However, in other realms, we have seen that assumptions based on findings from the US are not always true elsewhere. For example, in many places in Europe there has been a proliferation of news in prime time, while it is dwindling in the US ([14]), and news in the US is more strategy-focused than news in Europe ([15]). All in all this leads us to pursue a strikingly simple, but fundamental and necessary research question: to what extent do we find traces of PSE in a context that is dominated by a multiplicity of political parties and less political parallelism in the media system?

## Methods

The Ethical Board of the Amsterdam School of Communication Research (Universiteit van Amsterdam) approved of this study. Respondents provided their written consent to participate in the study.

To investigate this question we need a country characterized by a multi party system and low levels of political parallelism. We opt for the Netherlands, which is an interesting case in itself, representative of the democratic-corporatist model ([7]), fulfils our case selection criteria, and has seen a surge in the supply side of political information.

We make use of data from the European Election Campaign Study 2014 ([16], 2014; *N* = 2833), which was collected in the run up to the 2014 European Elections in collaboration with TNS NIPO, an international research agency. We use the first wave (fielded in December 2013), which include extensive background characteristics as well as a detailed program specific list of media exposure variables (see [17]). 3646 panel members of the TNS NIPO panel were invited to take part in this first wave (response rate = 77,7%). The sample is taken from the TNS NIPO Panel which contains around 200,000 Dutch households, representative of the Dutch population, and recruited using multiple strategies, mostly face to face and telephone recruitment. The sample by and large resembles the Dutch adult population with regard to gender, age, education, region, party choice at the Dutch Parliamentary Elections of 2012 ([16]).

Respondents were asked to indicate how many days in an average week they use several specific media outlets. Additionally, we tapped party preference of each respondent to see whether media outlets are selected along party lines, and asked respondents how much they are interested in politics on a scale from 1 to 7 (*M =* 3.93, *SD =* 1.70).

In all the analyses, we include 17 media outlets, among which the main public and commercial news and current affairs programs, the most used online sources, and several newspapers: the more right-leaning and tabloid style newspapers *Telegraaf* and *Algemeen Dagblad*, the elite newspapers *Volkskrant* and *NRC/nrc*.*next*, two free dailies, and regional newspapers. For reasons of parsimony, we only present the results for a selection of these news outlets, since outlets within the same category show similar results. Results for all outlets are available upon request, or can be found in [18] (The minimal data set underlying our results can be found in S1 File.)

In this Research Note we first map the average consumption of each source in the whole sample, and split out per group of partisans. This gives us a first indication of PSE, although it does not indicate whether adherents of a certain political party also have a similar media diet, distinct from adherents of a different party. This analysis also does not allow us to control for confounding factors.

In a next step we use a Latent Profile Analysis (LPA), a latent cluster analysis using scale variables instead of dichotomous items, to test whether there are clear profiles in media use. LPA “recovers hidden groups from observed data” ([19]). An LPA results in categorical latent variables that represent classes/profiles of individuals who share, in this case, similar media diets. The exposure to the 17 media outlets mentioned above are included as latent profile indicators (as well as two additional outlets), while gender, age, education, and party preference are included as covariates to predict membership to classes. (An analysis without these covariates leads to similar results.) Using Maximum Likelihood estimation, LPA uses all observations on the continuous indicators (in this case the media exposure variables) to define these classes. In LPA, the probability that a respondent belongs to one of the profiles is estimated simultaneously with the overall model. To determine the optimal number of profiles, similar models, only differing in numbers of classes/profiles, are estimated iteratively, and model fit indices are used to test which model fits the data best. The Bayesian Information Criterion (BIC) indicates which of the models is the most *parsimonious*, and the Lo–Mendell–Rubin likelihood ratio test (LMR LRT) compares the models and tests whether a model with less profiles fits the data better than the current model. The LPA indicated the 4-profiles-solution is most ideal. Even though the BIC decreased when more profiles were added, the LMR LRT indicated that the four group solution was preferred. The BIC is 205698.545 in the four group solution and the LMR LRT is 2915.260 (p = 0.240) in the five group solution. In this analysis, the four profile model therefore fits the data significantly better than the five profiles do ([20]). Moreover, entropy, which “measures the ability of a (…) model to provide well separated clusters” and for which values approaching one indicate clear delineation of classes ([21]), has a value of .942 in the four-profile solution.

In a third and final step, we identify the social and political profile of these groups with distinctive media use patterns, using multinomial regression. This allows us to decipher whether it is the case that respondents belonging to latent classes of media users are characterized by different political standings, controlling for their social background. A strong impact of partisan preference on membership of any of the profiles then indicates PSE: certain news is selected, based on partisan affinity, and other news is avoided, or rarely watched or read.

## Results

We first take a look at the average exposure to the most popular news and current affairs sources (Fig 1). The public broadcast news (*NOS Journaal*) and the commercial news show (*RTL Nieuws*–not shown here) are most watched: on average 3 days a week. More strikingly even: 75% of the respondents watch the *NOS Journaal* at least once a week, and 60% watch *RTL Nieuws* at least once a week. The second most popular news sources are regional newspapers (read on average twice a week), and online news sources. Current affairs and infotainment programs are typically watched once a week, and the different national newspapers are the least popular sources of information, though combined constitute a popular news source (see Fig 1 below).

**Fig 1:** Most popular News and Current Affairs Sources. For parsimonious reasons we only presented one outlet within the main television news categories. The results are similar for other outlets within the same category, and available from the authors upon request. Public News broadcast = *NOS Journaal*, Commercial news broadcast = *Hart van Nederland*, similar results for *RTL Nieuws*, Right-wing satirical news show = *Pownews*, Public Infotainment program = *DWDD*, Public current affairs program = *Nieuwsuur*, similar results for *Pauw & Witteman* and *EénVandaag*; Commercial talkshow = *RTL Late Night*; Free daily = *Metro*, similar results for *Sp*!*ts*; online news = *nu*.*nl*, similar results for newspapers online and “other news websites” Bars show exposure to each outlet in average number of days per week (Mean), error bars show standard deviation, labels show percentage of respondents indicating they use source at least once per week.

Table 1 shows the exposure to different media outlets among respondents preferring different political parties. In the table, one sample t-tests were used to test whether the average consumption within each party supporter group differed significantly from the sample average. We can discern some outlets that are more popular among right-wing populist voters (and among voters for *50Plus*: a party for senior voters with a populist twist): the commercial news broadcasts, the commercial talk show, and the tabloid newspaper *De Telegraaf*. And these outlets are much less used by those preferring the Greens. Some outlets are more popular among social democrats and social liberals, and at the same time less popular among right-wing populist voters, indicating a left-wing media diet: such as the public news broadcast, several current affairs programs, the public infotainment program, and the more left-wing newspaper de *Volkskrant*. But there are also many cross-cutting cleavages. For instance, voters for the liberal party, the social liberal party as well as Greens are readers of the quality newspaper *NRC*, and the current affairs program *Nieuwsuur* is popular among voters for mainstream parties and the niche party *50Plus* (not shown here). These results show some indication of PSE, but we proceed with the Latent Profile Analysis to investigate whether there are indeed distinct media diets.

**Table 1:** Exposure to news sources, related to party preference.

	Socialists	Greens	Soc-Dem	Social Liberals	Christ-Dem	Liberals	Right-Wing populists	Abstain	DK	Total
Public news broadcast	**3.60 (2.78)**	3.18 (2.60)	**3.87 (2.75)**	**3.78 (2.59)**	**4.48 (2.56)**	3.42 (2.66)	*2*.*73 (2*.*70)*	*2*.*27 (2*.*69)*	*2*.*63 (2*.*63)*	3.29 (2.74
	76,15%	80,52%	**81,97%**	**86,09%**	**89,78%**	**79,82%**	*66*,*67%*	*55*,*86%*	*66*,*13%*	74,69%
Commercial news broadcast	1.53 (2.17)	*0*.*97 (1*.*68)*	1.30 (2.12)	*0*.*92 (1*.*69)*	1.47 (2.10)	*1*.*25 (1*.*99)*	**2.27 (2.44)**	**2.00 (2.56)**	1.44 (2.13)	1.53 (2.20)
	47,40%	*36*,*36%*	*39*,*06%*	*34*,*21%*	47,11%	*41*,*28%*	**62,47%**	48,20%	46,64%	46,10%
Public Infotainment program	**1.91 (2.18)**	1.84 (2.12)	**1.97 (2.11)**	**2.00 (2.01)**	1.48 (1.93)	1.50 (1.85)	*1*.*14 (1*.*78)*	*1*.*13 (1*.*87)*	*1*.*29 (1*.*88)*	1.51 (1.97)
	**58,10%**	57,14%	**61,80%**	**64,29%**	50,22%	54,13%	*40*,*49%*	*36*,*49%*	*43*,*39%*	49,81%
Public current affairs program	**1.52 (1.94)**	1.49 (1.98)	**1.67 (2.02)**	**1.62 (2.02)**	**2.11 (2.24)**	1.40 (1.82)	*0*.*81 (1*.*64)*	*0*.*82 (1*.*74)*	*0*.*99 (1*.*71)*	1.31 (1.91)
	**51,68%**	49,35%	**55,79%**	**53,76%**	**63,56%**	**51,99%**	*28*,*89%*	*26*,*13%*	*34*,*80%*	44,48%
Commercial talkshow	1.03 (1.60)	*0*.*64 (1*.*28)*	0.98 (1.51)	1.09 (1.52)	0.97 (1.57)	1.09 (1.62)	**1.25 (1.88)**	0.91 (1.74)	1.10 (1.60)	1.05 (1.66)
	40,37%	*29*,*87%*	38,63%	**45,11%**	39,11%	42,20%	42,22%	*30*,*63%*	42,46%	39,64%
Satirical news show	0.51 (1.24)	0.34 (1.10)	0.48 (1.08)	*0*.*33 (0*.*92)*	0.42 (1.16)	0.46 (1.10)	**0.69 (1.45)**	*0*.*31 (0*.*93)*	*0*.*36 (0*.*94)*	0.45 (1.13)
	20,49%	*11*,*69%*	21,89%	16,54%	16,00%	21,10%	**25,43%**	*14*,*41%*	17,17%	18,92%
Telegraaf	0.85 (1.97)	*0*.*16 (0*.*71)*	*0*.*65 (1*.*70)*	0.86 (2.00)	1.02 (2.18)	**1.49 (2.52)**	**1.36 (2.37)**	0.90 (2.08)	0.90 (2.09)	0.99 (2.12)
	20,18%	*6*,*49%*	*17*,*17%*	19,92%	23,11%	**30,89%**	**31,36%**	20,27%	19,95%	22,56%
NRC/NEXT	0.15 (0.60)	**0.45 (0.11)**	0.28 (0.93)	**0.36 (0.98)**	0.19 (0.67)	**0.36 (1.06)**	*0*.*09 (0*.*48)*	*0*.*04 (0*.*31)*	*0*.*12 (0*.*56)*	0.20 (0.76)
	7,65%	**22,08%**	12,45%	**16,92%**	10,67%	**13,46%**	*4*,*94%*	*2*,*25%*	*5*,*80%*	9,07%
AD	0.83 (2.03)	0.57 (1.73)	0.89 (2.00)	0.69 (1.73)	0.95 (2.14)	0.80 (1.96)	0.88 (1.97)	*0*.*47 (1*.*48)*	*0*.*57 (1*.*61)*	0.76 (1.88)
	17,13%	11,69%	21,46%	17,29%	**22,22%**	17,43%	20,49%	*13*,*06%*	*14*,*39%*	17,58%
Volkskrant	0.51 (1.55)	**1.30 (2.36)**	**1.15 (2.25)**	**0.65 (1.75)**	0.40 (1.34)	0.36 (1.32)	*0*.*08 (0*.*46)*	*0*.*13 (0*.*66)*	*0*.*25 (1*.*13)*	0.41 (1.40)
	13,46%	**29,87%**	**26,61%**	**16,54%**	11,11%	9,17%	*3*,*95%*	*5*,*41%*	*6*,*26%*	10,66%
Free daily	0.47 (1.19)	0.60 (1.26)	0.60 (1.28)	0.45 (1.19)	*0*.*27 (0*.*85)*	0.40 (1.13)	**0.80 (1.62)**	0.52 (1.39)	0.40 (1.11)	0.49 (1.25)
	18,65%	27,27%	**24,03%**	18,05%	*12*,*44%*	15,90%	**26,67%**	17,57%	16,24%	18,78%
Regional Newspaper	2.40 (2.69)	2.03 (2.46)	2.28 (2.52)	2.33 (2.65)	**3.35 (2.66)**	2.03 (2.60)	*1*.*68 (2*.*25)*	*1*.*76 (2*.*36)*	*1*.*73 (2*.*46)*	2.12 (2.55)
	57,80%	54,55%	**61,37%**	58,65%	**77,78%**	*49*,*54%*	*49*,*88%*	*49*,*55%*	*46*,*17%*	55,35%
Online news	2.19 (2.74)	2.32 (2.64)	2.60 (2.71)	**3.03 (2.93)**	2.05 (2.66)	**2.82 (2.84)**	*1*.*88 (2*.*57)*	*1*.*54 (2*.*51)*	2.02 (2.64)	2.26 (2.73)
	50,76%	57,14%	**61,37%**	**62,78%**	48,44%	**61,47%**	*45*,*43%*	*35*,*14%*	48,49%	51,82%
N	327	77	233	266	225	327	405	222	431	

Entries in first row indicate average exposure to the source, in days per week, standard deviation in brackets. Entries in second row show percentage of respondents exposed to that specific source at least once per week. Bold numbers indicate significantly **more** consumption of that outlet within the party category, italic numbers indicate significantly *less* consumption; tested with one sample t-tests, p < 0.05. Small parties were included in the analysis, but left out of the table for parsimonuous reasons. Results available from the authors upon request. Liberals = *VVD*, social democrats = *PvdA*, right-wing populists = *PVV*, socialists = *SP*, christian democrats = *CDA*, social liberals = *D66*, Greens = *GroenLinks*.

Table 2 shows the results of the Latent Profile Analysis with the average media use per profile. The first group, the *minimalists*, uses the least media, but constitutes the largest group in the sample (65.94%) (This large group stayed intact, regardless of how many profiles were added to the analysis.) They watch the least (less than once a week) current affairs programs, barely read a newspaper, but do watch the public news broadcast or the commercial broadcast one to two days a week, and also follow the news online to the same extent. Even though these minimalists consume the least news and current affairs, we cannot say they completely *avoid* news.

**Table 2:** Media exposure per profile: average number of days per week.

	minimalists	public news consumers	popular news consumers	omnivores	Total
Public News broadcast	*2*.*33(2*.*42)*	**5.81 (1.84)**	3.39 (2.69)	**4.72 (2.48)**	3.29 (2.74)
	*66*.*0%*	**97.2%**	75.4%	**89.8%**	74.7%
Commercial News broadcast	1.49 (2.17)	**1.73 (2.30)**	**1.95 (2.30)**	*0*.*77 (1*.*63)*	1.53 (2.20)
	45.1%	**50.8%**	**57.1%**	*27*.*1%*	46.1%
Public infotainment program	*1*.*08 (1*.*64)*	**2.50 (2.30)**	1.77 (2.01)	**2.46 (2.29)**	1.51 (1.97)
	*41*.*2%*	**69.7%**	**57.1%**	**65.7%**	49.8%
Public current affairs program	*0*.*46 (0*.*92)*	**3.59 (2.01)**	1.26 (1.92)	**2.58 (2.19)**	1.31 (1.91)
	*26*.*8%*	**91.6%**	41.4%	**74.7%**	44.5%
Commercial talk show	*0*.*93 (1*.*53)*	**1.40 (1.91)**	1.29 (1.88)	0.90 (1.57)	1.05 (1.66)
	*37*.*0%*	**47.5%**	44.5%	34.3%	39.6%
Satirical news show	*0*.*26 (0*.*81)*	**0.87 (1.59)**	**0.77 (1.45)**	0.61 (1.32)	0.45 (1.13)
	*13*.*1%*	**32.1%**	**28.8%**	25.3%	18.9%
De Telegraaf	*0*.*83 (1*.*99)*	**1.27 (2.36)**	**1.38 (2.20)**	1.25 (2.31)	0.99 (2.12)
	*18*.*6%*	**28.6%**	**37.7%**	27.1%	22.6%
Algemeen Dagblad	*0*.*57 (1*.*66)*	**1.06 (2.23)**	**1.17 (2.09)**	**1.29 (2.26)**	0.76 (1.88)
	*13*.*2%*	**23.4%**	**31.9%**	**29.5%**	17.6%
de Volkskrant	*0*.*44 (0*.*27)*	*0*.*12 (0*.*42)*	*0*.*27 (0*.*77)*	**5.70 (1.13)**	0.41 (1.40)
	*3*.*2%*	*8*.*7%*	*12*.*6%*	**100%**	10.7%
NRC / nrc.nxt	*0*.*10 (0*.*53)*	**0.29 (0.88)**	0.26 (0.83)	**0.89 (1.55)**	0.20 (0.76)
	*4*.*9%*	**13.7%**	12.0%	**35.5%**	9.1%
Free daily	*0*.*18 (0*.*54)*	*0*.*18 (0*.*53)*	**4.34 (1.20)**	**0.72 (1.48)**	0.49 (1.25)
	*11*.*9%*	*12*.*2%*	**99.5%**	**27.7%**	18.8%
Regional newspaper	*1*.*74 (2*.*38)*	**3.25 (2.75)**	2.03 (2.32)	2.43 (2.56)	2.12 (2.55)
	*48*.*3%*	**72.4%**	**62.8%**	**63.3%**	55.3%
Online news	2.19 (2.74)	2.28 (2.67)	2.44 (2.70)	**2.81 (2.88)**	2.26 (2.73)
	49.9%	53.6%	57.1%	**60.2%**	51.8%

First row: Average number of days per week in cells; standard deviations in parentheses. Second row: percentage of respondents in profile that is exposed to the source at least once per week. Bold numbers indicate a higher use than the sample average, italic numbers indicate lesser usage than the sample average; tested with one sample t-tests, p < 0.05.

The second group of media users is much smaller (21.46% of the sample) and can be characterized as *public news consumers*. The public news broadcast is missed only once per week, and these people most often watch current affairs programs: they watch two of the main programs every other day. They read the popular newspapers *De Telegraaf* and *Algemeen Dagblad* once a week.

The third group is small (6.74% of the sample) and can be discerned by watching news on commercial channels most often. These *popular news consumers* also are very fond of free newspapers (they read them four days a week) and the most avid readers of the popular newspaper *De Telegraaf*.

The final, also small, group of media consumers (5.86% of the sample) we define as *omnivores*. They are exposed to all news and current affairs media at least once a week. Additionally, they are characterized by reading de *Volkskrant* and the *NRC* or *nrc*.*next*. Finally, they watch the public news broadcast relatively often and most often use online news media. Even though these omnivores use more “left-wing media” than the media users in the other profiles do, and watch commercial programs, popular among right-wing populist voters, much less, we cannot say this profile is the left-wing profile, as these omnivores also read the more right-wing *De Telegraaf*.

Other patterns attract our attention too. First of all, respondents within all profiles consume online news at least twice a week, which does not indicate a digital media gap. However, it has to be noted that only half of the respondents go online to consume news. The same holds for watching news broadcasts. Especially the public news broadcast stands out: in Fig 1. we saw this is the most popular news source, and in Table 2 it becomes clear that it plays a central role in each media diet: it is always more popular than the other two news broadcasts (not shown here). Other news sources are much more differentiating. For instance, only public news consumers and omnivores often watch current affairs programs, and only omnivores read de *Volkskrant* and the *NRC*, while the free dailies are mostly read by popular news consumers. The public news broadcast is watched at least once a week by 66% of the most avid news avoiders (the minimalists), for whom it is their most important news source. Overall, these results show that Dutch news consumers indeed selectively expose themselves to certain news content, and also avoid news content. However, it is thus far unclear whether this selectivity is based on political (dis)agreement.

In a final step we therefore focus on what characterises the media consumers of these different diets. Table 3 shows the results of a multinomial logistic regression analysis in which the membership of each group is predicted using social background characteristics, political interest, and party preference. The minimalists are the reference category.

**Table 3:** Predictors of media profiles, multinomial regression analysis with minimalists as reference category (unstandardized regression coefficients).

	Public news consumers	Popular news consumers	Omnivores
Gender	-0.05	-0.30	-0.23
Age	0.06***	-0.01*	0.03***
Education	0.01	-0.12*	0.37***
Political Interest	0.43***	0.18***	0.54***
Socialists	0.14	0.28	0.52
Greens	-0.18	0.73	1.25*
Social democrats	-0.13	0.70*	1.11**
Social liberals	-0.05	0.27	0.15
Christian democrats	-0.25	0.01	-0.26
Liberals	-0.13	-0.03	-0.32
Right-wing populists	-0.19	0.84**	-1.91*
Non-voters	-0.13	0.48	-0.99
Constant	-5.91***	-1.93**	-8.05***
Log Likelihood	-2245.18		
Pseudo explained variance	16.84%		

* = p > 0.05

** = p > 0.01

*** = p > 0.001. Coefficients for the small Christian parties, Animal Party, and Senior Party (50Plus) not shown here; n = 2833.

It becomes clear that the groups differ in social background. Public news consumers and omnivores are older as well as higher educated, compared to the minimalists. The popular news consumers are more often female and lower educated. So we do see four specific clusters with regards to the social profile. Additionally, there are differences between the profiles with regard to their political interest. Public news consumers, compared to minimalists, are more interested in politics (measured with the item: ‘How interested would you say you are in politics?’: scale from 1 (not at all interested) to 7 (very interested)). This also holds true for popular news consumers, but to a lesser extent. The minimalists thus can be distinguished by their low political interest.

The multinomial regression, finally, checks whether the groups differ from each other in political preference, with respondents with no particular preference as the reference category. Public news consumers do not differ from minimalists, but popular news consumers and omnivores do. Popular news consumers more often prefer (the very different) social democrats and the right-wing populist party. Among omnivores we also find more social democrats, but significantly less right-wing populist voters. Additionally, we find many Greens holding a media junkie diet. The results do not indicate a clear right-wing profile, whereas the omnivores diet could be indicated as somewhat leftist. (Note that if we include ideology as a predictor, we find that public news consumers and omnivores are significantly more left-wing than minimalists.) Overall, these results indicate there is some evidence of PSE in the Netherlands.

## Discussion

This research note examined to what extent traces of PSE can be found in a non-US context that is rather dominated by a multiplicity of political parties and a different configuration of the media system. This is a rather fundamental question, as we should not necessarily assume that the patterns and consequences of news consumption travel across systems. Our results show some important insights. In general and using descriptive data, we found that citizens preferring specific political parties did differ in their exposure to certain media outlets. It seems that many left-wing voters prefer public news and current affairs programs and the left-wing elite newspaper de *Volkskrant*, while right-wing populist voters favoured the right-leaning, tabloid style newspaper de *Telegraaf*, the popular news broadcast and a satirical news show. Such specific patterns corroborate with findings of [8], and show that Dutch news consumers with different political party preferences do have somewhat different media diets. Although we did not find a completely polarized picture (which is certainly more present in the US), this is an indication of partisan press relations and parallelism.

These findings became also evident when we examined specific media profiles. Four profiles in media use were distinguished: A large group, the minimalists (65.94%), a smaller group, the *public news consumers* (21.46%), and two very small groups, *popular news consumers* and *omnivores* (6.74% and 5.86%, respectively). Moreover, we found that minimalists are less interested in politics than people who are more often exposed to mass mediated news and information. With regard to political preferences, public news consumers do not differ from minimalists, but the popular news consumers and omnivores do. Popular news consumers are more likely to vote for the Social Democrats, as well as the Right-Wing Populists. Yet, omnivores are more likely to vote for the Social Democrats and the Greens, and less likely to vote for the Right-Wing Populists. Interestingly, not one specific group of citizens simply ignored (all) political information, indicating ‘selective avoidance’: the practice of screening out counter-attitudinal information ([22]). Even though we see that right-wing populist voters seem to opt out of the ‘omnivores’ diet, the latent profile analysis also shows that many news sources reoccur in the different media diets. Consequently, also the minimalists, albeit limited, consume news.

We interpret the minimalists–the largest group–as representing a *quasi-monitorial citizen*. This is derived from the concept *monitorial citizens* introduced by [23]. He suggested that in the US, a group of politically interested citizens exists, that sporadically consumes news, because they have other interests as well. As minimalists are not the most politically interested citizens, they still seem to consume media to get an overview of political news. Additionally, and contrary to our expectations, this study did not find two completely separate ideological camps with matching media diets as has been found in the US context (see e.g., [8]). Still, we found some evidence that left-wing oriented voters are more likely to consume a more extensive media diet, while right-wing voters are more likely to prefer commercial and popular news. Collectively, these findings help us to understand the types of information different citizens are exposed to.

Looking ahead in a rapidly changing media environment, we propose two optimistic viewpoints. First of all, in particular in terms of social media, [24] suggest that the context of choice of stories is different and that social cues play a role such that social endorsements provide a cue that suggests utility of news, which can overcome PSE processes. Second, and more importantly, the findings show that the public news broadcast is not only the most consumed news program, but it is also the most often used news source for individuals within the different profiles. Even though Dutch citizens indeed expose themselves to different media, in part based on partisan affiliation, members of none of the clusters completely avoid the public broadcasting news because of expected disagreement. This is entirely different compared to the US, where public broadcasting plays a marginal role; it only reaches a minimum amount of US citizens. In the Netherlands, the public news broadcast can be found in each of the four media profiles, and plays the lead role in the minimalist media diet. This suggests that it plays a unifying, and nation-binding role in this fragmented media landscape with an abundance of choice. In the Dutch situation, a solid public broadcaster, with, in particular, a strong public news provision, is an important condition to avoid the US situation where the public sphere appears to have become different public spheres.

## Supporting Information

S1 File Minimal data set underlying results. This is the minimal data set underlying the results in this study. It includes an id variable, background characteristics (gender, age, education, political interest, vote choice if elections were held tomorrow) media exposure to 19 sources in days per week, dichotomous variables for party preferences, and the media profiles the respondents were assigned to based on the latent profile analysis.
(DTA)
